# Multi-Flexible Body Dynamics Modeling and Experimental Study of the Patient Rehabilitation Transfer Device

**DOI:** 10.1155/2022/6610753

**Published:** 2022-10-14

**Authors:** Wu Ren, Kailu Zhang, Xueling Zhang, Ziya Zhao, Fei Lin, Kai Xie, Jia Li, Yi Yu

**Affiliations:** ^1^Xinxiang Medical University, School of Medical Engineering, Engineering Technology Research Center of Neuroscience and Control of Henan Province, Xinxiang Engineering Technology Research Center of Intelligent Rehabilitation Equipment, Xinxiang, Henan 453003, China; ^2^The First Affiliated Hospital of Xinxiang Medical University, No. 88, Health Road, Weihui Xinxiang, Henan 453100, China

## Abstract

**Objectives:**

The patient rehabilitation transfer device is a typical personnel transfer equipment, which is mainly composed of outriggers, support arm, lifting arms, hooks, handrails, hydraulic cylinders, and other components. The existing research on the device is mainly focused on the configuration design and transfer mode, and the research on its dynamic characteristics during the transfer process has not been thoroughly discussed. *Methodology*. Based on the existing research, a portable hydraulic rehabilitation patient transfer device has been developed. Then the multi-rigid body dynamic and finite element flexible body models were established. Next, the dynamic characteristic difference between the two models of the device was studied.

**Results:**

As shown in the results, the finite element multi-flexible body model has obvious flexible vibration in the lifting stage, and the amplitude reaches 16 mm in the motion startup stage due to the influence of rigid-flexible coupling. The tip acceleration of the flexible body model was also influenced by the vibration, and the maximum acceleration value reaches 0.06 m/s^2^. According to the test results, the maximum acceleration of the terminal reaches 0.05 m/s^2^, which is close to the finite-element multi-flexible model simulation results. The experimentally measured natural frequency of the device is 3.1 Hz, which is also close to 3.2 Hz calculated by the simulation. Because the flexible component in the flexible model is only the lift arm, the natural frequency is slightly larger than the experimental value.

**Conclusion:**

According to the stress value of the finite element multi-body model motion process, the maximum stress appears at the moment when the motion reaches the top end, and the instantaneous stress reaches 206 Mpa, which is in line with the allowable stress range of the material design. The data obtained in this study will provide help for the follow-up clinical rehabilitation and intelligent device research.

## 1. Introduction

Aging and disease can lead to decreased muscle strength in the lower extremities, causing some difficulty for older adults and patients to stand and walk. Rehabilitation and Special Equipment for Disabled Persons organized a review meeting on the standard of wheelchair vans, and National Research Center for Rehabilitation Technical Aids also carried out the drafting of the corresponding standard in 2015. The National Standardization Administration Committee released “requirements and test methods for lifts for the dysfunctional” to provide guidelines for the development of related standards in 2020. The device can solve the problem of the movement of the elderly and patients in the daily activity area to a certain extent. However, the degree of automation and market promotion of mobility aids in China is still low, and there is still a gap between the economy and its applicability to developed countries.

## 2. Literature Review

The main research on assistive rehabilitation lifting devices at this stage was mainly as follows: Kulich et al. [1] designed the AgileLife patient transfer system, which effectively improves mobility maneuverability for people with disabilities and their families and caregivers. Tongbo et al. [2] studied the difference and connection between the contact stress on the articular surface cartilage of the two modes of rearfoot strike and non-rearfoot strike, which helped the study of human gait balance. Caidong et al. [3] used the ATmega128 controller to study the motion stability of the hanger of a patient lift. In the same year, Greenhalgh [4] did a study on tension, mobility, and cognitive load during human transfer to reduce the physical discomfort of the personnel involved and improve the use of the human-machine interface. Wu [5] designed a transfer robot capable of assisting people to stand and reduce the muscle strength of the patient's lower limbs. An assistive lift robot designed by Koyama [6] is easier to enhance the independence of patients and reduces the cost of caregivers. Lin [7] investigated and analyzed the effect of different patient lifts using a robot simulating actual patients and made more comparisons in terms of patient rehabilitation training. Benoit et al. [8] investigated the countermeasure method of manual lift in transferring overweight patients and made improvements in related equipment devices, and Humphreys [9] designed a transfer aid in which patients can use a force-sensing handle for speed control, reducing the amount of caregiver labor while greatly increasing the automation of the related equipment. Mombaur [10] used a simulation approach to achieve the prediction of stable motion in elderly subjects. The approach has been used in the modeling of human multibody system to achieve dynamics and investigate different support forces in the human body now. In the same year, Sun et al. [11] used four different sliding mobility devices to achieve wheelchair to bed and bed to wheelchair transfer of patients and compared the range of different sliding devices. Based on ergonomic principles, Nodooshan [12] developed an assistive device to increase the comfort of the user and operator and reduce the user's physical exertion and single working posture. By using the ultrasonic principle, Humphreys [13] developed an impedance-controlled patient transfer aid with force feedback so that the lift can better avoid obstacles during the movement. Based on vibration compensation methods, a biomechanical dynamics model has been established by Humphreys et al. [14] and in which human–machine comfort had been studied which effectively reduce the vibration of related equipment.

In summary, most of the existing studies on lifting devices at home and abroad have focused on the development and improvement of device types and the convenience of personnel operation, the study of the dynamics of the multi-flexible body dynamics of patient rehabilitation lifts with rigid-flexible models has not been reported till now. So far, the two main approaches for the dynamic modeling of elastic robotic manipulators have been the finite element method (FEM) and the assumed mode method (AMM). AMM is a powerful method that provides the link's deflection at each point [18–21, 25, 26]. Usoro and Heidari, respectively, put forward different finite element modeling methods for flexible body linkage [22–24]. In this study, the multi-flexible body model of the common manual hydraulically driven patient rehabilitation transfer device had been established by the finite element method and virtual spring damping method. In the model, the flexible lifting arm and the driving cylinder were, respectively, equivalent to the flexible body, and then the law of mechanical characteristics such as end displacement, hydraulic cylinder force, and inherent frequency with time for both models had been discussed. Next by using the existing dynamic signal acquisition machine, a test was executed; the accuracy of the model was verified then. And the results and conclusions obtained can assist the development of relevant medical rehabilitation equipment products and provide some data support in the integration of engineering and clinical aspects.

## 3. Multi-Body Modeling of the Patient Transfer Device

### 3.1. Virtual Spring Damping Method of Lifting Cylinder

The lifting arm of the transfer device is driven by hydraulic cylinder. In this model, the virtual spring damping method was used to simulate the hydraulic cylinder with certain stiffness and damping, which is used to control the movement of the hydraulic cylinder. The equivalent spring damping of the driving cylinder and the connection of the lifting arm [15] are shown in Figure 1.

The lifting cylinder is the driving device, according to the hydraulic cylinder equivalent method, the force *F*_cy1_ and motion displacement *y* of the equation of motion can be expressed as follows:

(1) $$\begin{array}{c} F_{\text{cy}1}=k\cdot \left(y_{0}\left(t\right)-y_{\text{cyl}}\left(t\right)\right)+c\cdot {\left(y_{0}\left(t\right)-y_{\text{cyl}}\left(t\right)\right)}^{\prime }, \end{array}$$

(2) $$\begin{array}{c} y=\int_{t_{0}}^{t}-\frac{F_{\text{cyl}}-k\left(y_{0}\left(t\right)-y_{\text{cyl}}\left(t\right)\right)}{c}\text{d}t, \end{array}$$

(3) $$\begin{array}{c} c=\frac{\pi \eta {ld}^{2}}{{\left(D-d\right)}^{2}}\left[3+\frac{3d}{4\left(D-d\right)}\right]. \end{array}$$

In equation (1) and (2), *y*_0_(*t*) is the initial position of the lifting cylinder, and *y*_cy1_(*t*) is its motion termination position, and *t* is the lifting motion time. In this simulation model the device is driven by the driving cylinder motion displacement. Then the device force magnitude over time trend can be analyzed. In equation (3), *c* is the hydraulic cylinder damping, *l* is the piston length, and *d* is the piston inner diameter, *D* is the cylinder inner diameter, *η* is the hydraulic oil viscosity. According to the existed prototype hydraulic cylinder parameters, the equivalent value of the driving cylinder damping in this simulation model is 0.01 N · S/mm. By using the series–parallel relationship of the cylinder spring damping method, the equivalent stiffness of the cylinder was calculated as 3 kN/mm.

### 3.2. Finite Element Multi-Flexible Body Modeling

In the augmented formulation, the method of Lagrange multipliers that can be applied to both holonomic and nonholonomic systems is used. The rigid body motion equation [16, 17] of multibody system can be expressed by the following formula (4):

(4) $$\begin{array}{c} F=B^{T}\left(M\overset{•}{Y}+\Phi_{Z}^{T}\lambda -Q\right)=0. \end{array}$$

In equation (4), *Φ* are joint constraints and *λ* = [*λ*_1_*λ*_2_ ⋯ *λ*_*nc*_]^*T*^ is the vector of Lagrange multipliers. *M* is the mass matrix, and *Q* is the external force vector in the included Cartesian coordinate system.

The rigid body motion equations can be further extended from equation (4) and then equation (5) can be obtained:

(5) $$\begin{array}{c} F^{r}=B^{T}\left(M\overset{•}{Y}+\Phi_{Z}^{\text{rr}T}\lambda^{\text{rr}}+\Phi_{Z}^{\text{er}T}\lambda^{\text{er}}-Q^{r}\right)=0. \end{array}$$

In equation (5), the superscript *r* represents the number of rigid bodies, the superscript rr represents the number of rigid bodies between each other, and the superscript er represents the number between flexible body nodes and rigid bodies. The constraint equation between rigid bodies can be expressed as a function of the generalized coordinates *q^r^* of the rigid bodies as in equation (6):

(6) $$\begin{array}{c} \Phi^{\text{rr}}=\Phi^{\text{rr}}\left(q^{r},t\right). \end{array}$$

Similarly, the motion equation of the flexible body can be derived as formula (7):

(7) $$\begin{array}{c} F^{e}=M^{e}{\ddot{q}}^{e}+\Phi_{q^{e}}^{\text{ee}T}\lambda^{\text{ee}}+\Phi_{q^{e}}^{\text{er}T}\lambda^{\text{er}}-Q^{e}=0. \end{array}$$

In equation (7), the superscript *e* stands for the number of flexible body nodes, and *q^e^* is the generalized coordinate of the flexible body nodes. The superscripts ee stands for the number of flexible nodal bodies between each other, and the superscripts er indicate the number of flexible body nodes and rigid bodies between each other. The forces *Q^e^* between the flexible body nodes can be expressed as the sum of the forces between the elements and the applied forces (e.g., gravity or contact forces) as equation (8):

(8) $$\begin{array}{c} Q^{e}=Q^{\text{element}}+Q^{\text{applied}}. \end{array}$$

The joint constraint between the flexible body node and the virtual rigid body can be expressed as equation (9):

(9) $$\begin{array}{c} \Phi^{\text{er}}=\Phi^{er}\left(q^{e},q^{r},t\right). \end{array}$$

Similarly, the constraint equation between the nodes of the flexible body can be expressed as equation (10):

(10) $$\begin{array}{c} \Phi^{\text{ee}}=\Phi^{\text{ee}}\left(q^{e},t\right). \end{array}$$

Therefore, the finite element flexible multibody (MFBD) system matrix can be expressed by equation (11) and can be solved by the augmented sparse matrix solver.

(11) $$\begin{array}{c} \left[\begin{array}{ccccc} \frac{\partial F^{e}}{\partial q^{e}} & \Phi_{q^{e}}^{\text{ee}T} & \frac{\partial F^{e}}{\partial q^{r}} & 0 & \Phi_{q^{e}}^{\text{er}T}\\ \Phi_{q^{e}}^{\text{ee}} & 0 & 0 & 0 & 0\\ \frac{\partial F^{r}}{\partial q^{e}} & 0 & \frac{\partial F^{r}}{\partial q^{r}} & B^{T}\Phi_{Z}^{\text{rr}T} & B^{T}\Phi_{Z}^{\text{er}T}\\ 0 & 0 & \Phi_{q^{r}}^{\text{rr}} & 0 & 0\\ \Phi_{q^{e}}^{\text{er}} & 0 & \Phi_{q^{r}}^{\text{er}} & 0 & 0 \end{array}\right]\left[\begin{array}{c} \Delta q^{\text{ee}}\\ \Delta \lambda^{\text{ee}}\\ \Delta q^{\text{rr}}\\ \Delta \lambda^{\text{rr}}\\ \Delta \lambda^{\text{er}} \end{array}\right]=-\left[\begin{array}{c} F^{e}\\ \Phi^{\text{ee}}\\ F^{r}\\ \Phi^{\text{rr}}\\ \Phi^{\text{er}} \end{array}\right]. \end{array}$$

Equation (11) is a system of differential equations of motion that along with the constraint equations can be solved for the vector of system generalized coordinates *q* and the vector of Lagrange multipliers *λ*. This equation is used as the basis for developing many general computational algorithms for the dynamic analysis of multibody systems subject to both holonomic and nonholonomic constraints [26].

As can be seen above, although the finite element multi-flexible body method is used to describe the deformation of the structure by the relative displacement and rotation as node coordinates which has high computational accuracy, the scale of the system solution is large and the efficiency of solving is relatively low. But it can be used for systems with relatively simple components and a relatively small number of unit nodes and high solution accuracy requirements.

### 3.3. Physical Model of the Transfer Device

The simulation model of the hydraulic lift was established with the following assumptions in this study:

(1) Only calculate the kinematics and dynamics of the transfer device in the positive plane of the lifting and pushing patient, and ignore the effect of the possible left and right torsion of the transfer device on the dynamic characteristics. The lifting arm is equivalent to flexible body, the other connecting rods are still equivalent to rigid bodies due to the actual work.

(2) The connection between the vertical arm, the support arm, the swing arm, and the hanger is equivalent to the revolute and fixed joint, and the driving of the lifting hydraulic cylinder is equivalent to the translational joint.

Due to the characteristics of this prototype, the movement speed of the driving cylinder and the boom is relatively small, so the effect of simulated Coriolis and centrifugal acceleration on the transfer device operation has been neglected.

Based on the above rules and the actual device structure, a diagram of a rigid body and the finite element multi-flexible models of the patient rehabilitation transfer device are as shown in Figure 2.

The number of supporting arms, vertical arms, lifting arms, hooks, and kinematic pair types in the equivalent model are as shown in Table 1.

## 4. Simulation and Experimental Verification

### 4.1. Simulation Model

According to the basic theory and assumptions, the actual operation situation has also been considered. The rigid body motion model of the transfer device was established in RecurDyn software. In the model, the supporting wheels and vertical arm were fixed on the outriggers. The vertical arm was connected to the lifting frame through the cylinder, the handrail and the vertical arm were connected by a fixed joint, and the end of the lifting frame was connected with the hook and the personnel sling. The basic parameters of the rigid body model and the main components are shown in Table 2.

In Table 2, the lifting arm size is the straight-line distance from the start point to the end point. According to the previous finite element flexibility scheme, the lifting arm, which has the greatest influence on the apparatus motion, was subjected to finite element flexibility. Other parts were treated as rigid bodies due to the small flexibility influence. This will reduce the calculation scale and improve the calculation efficiency. After that, the finite element multi-flexible body model was established, and the spring damping system for driving the cylinder was established by the virtual spring damping method also. After the rigid body model and the finite element multi-flexible body model of the transfer device was established, the working conditions of the transfer device were simulated by lifting and transferring patient, and the vibration law, cylinder force, lifting boom stress and tip displacement during the motion of the two models were analyzed then which can be help for the improvement of the comfort and safety design of the device.

### 4.2. Result Analysis

According to the above papers and research assumptions, the rigid body motion model and the finite element multi-flexible body model of the device were established in RecurDyn software then as shown in Figure 3. The motion was controlled by the step function to control the stroke of the hydraulic cylinder. The stress distribution of the patient during lifting and forward movement simulated by the finite element flexible body model is shown in Figure 4(b). In Figure 4, the motion acceleration and stress of the device are relatively large in the three stages of the lifting, initial stage of horizontal motion, and the termination stage, which conforms to the change in actual working conditions. To correspond to the subsequent experiments, a concentrated mass of 55 kg was added at the end of the transfer device to simulate the mass of the human body. The fflex module of RecurDyn software was used for simulation. The MFBD (Multi flexible body dynamics technology) inside the module was adopted to connect the rigid multi-body system with the finite element flexible body. They were connected through the common rigid region as shown in Figure 4(a), and then the relevant motion pairs were defined in the solving process. The fflex module in RecurDyn can be used to directly perform finite element meshing of the lifting arm. The efficiency and speed of the solution were taken into account in this study either. The finite element meshing of the lifting arm was adopted as automatic size, as shown in Figure 4(b) (total 17,661 elements, 8824 nodes, and the element type was the tetrahedral element). According to the calculation results from RecurDyn professional and flexible module it could be concluded that the maximum stress value during the motion of the device was 206 Mpa as shown in Figure 4(b), which was located at the joint of the hydraulic drive cylinder and the lifting arm, and the stress values in the lifting stage and the initial stage were higher during the motion process. The maximum stress value occurred near the end time of the motion. With the motion near the stopped time the flexible lifting arm vibration also attenuation and the stress also decreases accordingly. Under the simulated lifting operating conditions. The change was always within the allowable stress of the boom material Q345B (a kind of steel, and its material yield value is about 345 Mpa).

### 4.3. Simulation Research on Boom Tip Displacement

In Figure 5, the rigid body model of the transfer device was moved relatively smoothly during lifting, while the finite element multi-flexible body model had flexible vibration during the motion. And the amplitude of the flexible vibration reached 16 mm during the time of starting, which better shown the characteristics of the flexible characteristic of the transfer device.

### 4.4. The Force of Lifting Cylinder Research

The cylinder force changes of the two models could be concluded from Figure 6: the force change of the oil cylinder of the rigid body model was small. After the force changed to a certain extent in the lifting and horizontal motion states, the force was stable until the end of the movement, and finally reached 1650 N. However, because of the obvious flexible vibration influence of the finite element multi-flexible body, the force of the cylinder had also showed a strong change rule. Especially, there was a flexible change in the initial stage of lifting, and finally the force of the cylinder reached 2903 N, which was about 1.5 times the maximum force of the rigid body model, and was closer to the actual working situation. Therefore, when the transfer device prototype needed to be improved, the considering of finite element multi-body calculation results of cylinder force is needed. The maximum force of the hydraulic cylinder of the two models changed with time is as shown in Table 3.

### 4.5. Experimental Studies and Results Discussion

To verify the simulation analysis results, an experiment was conducted by using Dewesoft 32-channel dynamic strain gathering analyzer, a three-axis acceleration sensor, an inclination sensor (Figure 7), and a transfer device prototype. The instrument connection and personnel riding diagram (personnel mass 55 kg, corresponding to the simulation above) were as shown in Figure 8. To simulate the finite element multi-flexible body model to the maximum extent, the motion rule between the simulation one and the experimental operation were same. In the test the corresponding motion drive was obtained by manipulating the lifting cylinder. The terminal acceleration signal was as follows in Figure 9. Through the analysis of the terminal acceleration signal, it could be concluded that the natural frequency of the transfer device added with passenger was 3.1 Hz. The displacement of the cylinder at the starting position in the experiment was at 15 cm, and the cylinder moved 1 cm of the pressure rod in one stroke, and the person started to lift at 31 cm position. The maximum displacement of the cylinder was 46 cm, and then the translational motion had been executed and the final distance is about 2 m. And the flexible vibration existed at the end of the stopping process due to the flexibility influence.

The comparison of the tip maximum acceleration of the device test and the finite element multi-flexible body model is shown in Table 4. Due to the influence of flexible vibration, the maximum value reached 0.06 m/s^2^. According to the test data, the maximum acceleration of the transfer device was 0.5 m/s^2^, which was similar to the result of the flexible model, and the vibration trend of them was similar too. The tip acceleration difference between the test and flexible may be caused by the stiffness calculation deviation of the cylinder equivalent by spring damping method. Another reason is that in the simulation, only the lifting arm was equivalent to flexible body and other components were still equivalent to a rigid body.

In Table 5, the transfer device first order natural frequencies of the finite element multi-flexible body model and the measurement were 3.2 and 3.1 Hz. Because the lifting boom in the simulation model was a flexible body and the other connections and structures were still rigid bodies, the natural frequency was slightly higher than the actual prototype, which is consistent with the modeling characteristics. In addition, since the frequency of the main organs of human body is mostly higher than 3 Hz, the human body main organ's natural frequency resonance influence was avoided. Thus, the human riding discomfort was minimized.

## 5. Conclusion

A multi-rigid body model and a finite element flexible body model of a patient rehabilitation transfer device were established in this study, and their kinematics and dynamics characteristic were analyzed then. Next, the corresponding experimental comparison was carried out based on the existing device. The following conclusions can be drawn:

1. The rigid body model of the device was established first. To solve the equivalent problem of driving hydraulic cylinder, the virtual spring damping method were further used to establish the finite element multi-flexible body model.
2. The characteristic analysis of stress and displacement during the motion process of the device had been compared between the rigid and the flexible body model. Then the driving cylinder force, boom tip acceleration, and frequency had been discussed.
3. A test was carried out and the results were in good agreement with the simulation model, which proved the accuracy and necessity of the flexible body analysis and driving cylinder equivalence of the transfer device. This provided help for the subsequent transfer device prototype improvement and personnel comfort study.

Because of the inadequacy of the existing laboratory limitation, there is still deficiency in this research, and the future study can be strengthened in the following points:

1. To get better simulation effect, the finite element multi-flexible body modeling can further consider the other components with greater flexibility.
2. Lifting and forward motion were mainly focused one in this study without considering the influence of the left and right sway when a person is riding on the device. For a more practical study of the ride dynamics, the effect of the left and right sway can be considered in subsequent studies.

## Figures and Tables

**Figure 1:** Physical model of patient transfer device hydraulic cylinder.

**Figure 2:** Flow chart of patient transfer device dynamics modeling.

**Figure 3:** The patient transfer device multi-rigid body model is as shown in Figure3(a); the finite element meshing of lifting arm is as shown in Figure3(b); and the multi-flexible model is as shown in Figure3(c).

**Figure 4:** The rigid-flex connection rigid region is as shown in Figure4(a) and the stress coutor of the patient rehabilitation transfer device is as shown in Figure4(b).

**Figure 5:** Patient transfer device tip displacement of different models.

**Figure 6:** Hydraulic cylinder force comparison between the two models.

**Figure 7:** 32-Channel Dewesoft dynamic signal test acquisition and processing instrument.

**Figure 8:** Dynamic mechanical signal experiment of existing patient transfer device prototype.

**Figure 9:** Tip acceleration test curve of the patient transfer device.

**Table 1:** Equivalent connection of patient transfer device dynamics model.

	Model type	Number
Flexible body	Lifting frame	1
Rigid body	Pole, walking frame, hanger, support frame, handrail	8
Revolute joint	Stand, support frame, lifting frame, hanger, walking frame	8
Translational joint	Hydraulic cylinder and piston, traveling	2
Spring damper	Hydraulic cylinder	1

**Table 2:** Main parameters of the patient transfer device.

	Handrail	Bracket	Standing arm	Boom	Hydraulic cylinder
Size (mm)	329	1266	1104	919	450
Quality (kg)	1.6	13.54	20.15	2.82	4.45

**Table 3:** Hydraulic cylinder maximum force comparison between the two models (N).

The maximum force of the cylinder	Rigid-body model	Finite element multi-flexible body model
Lifting cylinder	1905	2903

**Table 4:** Maximum tip acceleration comparison between simulation and experiment (m/s^2^).

Finite element flexible body model	Fest value
0.06	0.05

**Table 5:** Natural frequencies between the simulation model and experiment data (Hz).

	Finite element flexible body model	Test value
Frequency	3.2	3.1

## Data Availability

The data used to support the findings of this study are available from the corresponding author upon request.
